# Prognostic Implication of a Cuproptosis-Related miRNA Signature in Hepatocellular Carcinoma

**DOI:** 10.1155/2022/4694323

**Published:** 2022-09-13

**Authors:** Ze Jin, Mengmeng Wang, Yajun Meng, Di Chen, Yushuang Xu, Xin Jiang, Zhifan Xiong

**Affiliations:** Department of Gastroenterology, Liyuan Hospital, Tongji Medical College, Huazhong University of Science and Technology, Wuhan, China

## Abstract

**Background:**

Hepatocellular carcinoma (HCC) is one of the most frequently diagnosed malignancies globally, accounting for the third cause of cancer mortality. Cuproptosis, a copper-induced cell death, was recently reported in *Science*. The purpose of this study was to evaluate the prognostic implication of cuproptosis-related miRNAs (CRMs) in HCC.

**Methods:**

Transcriptomic data and clinicopathological features of patients with HCC were extracted from the Cancer Genome Atlas (TCGA) database. Prognostic CRM signature was established by utilizing univariate Cox regression and LASSO analyses. To validate the accuracy of prediction, the Kaplan-Meier (K-M) and time-dependent receiver operating characteristic (ROC) analyses were adopted. A nomogram comprising clinical characteristics and the miRNA signature was developed to improve the prediction of patient outcomes. Finally, functional enrichment analysis and immune infiltration analysis were carried out.

**Results:**

Of CRMs, 14 were obtained to construct a prognostic miRNA signature. This CRM signature was an independent factor for predicting overall survival (OS). Kaplan-Meier curves demonstrated a noteworthy difference in survival rates between different risk subgroups (*p* < 0.001). The robust prognostic capacity of this signature was exhibited by sampling verification and stratified survival analysis. Functional analysis indicated that the high-risk group was mainly enriched in signaling pathways and different levels of immune infiltration were revealed between the two risk groups. The potential interaction of the model with the immune checkpoint activities was also detected.

**Conclusion:**

The CRM signature could act as an independent predictor to guide individual treatment strategies, which could provide fundamental insights for further studies.

## 1. Introduction

Liver cancer is the sixth most common cancer with almost 906,000 new cases in 2020, which ranks the third leading cause of cancer-related death worldwide [1]. Hepatocellular carcinoma (HCC) is the most prevalent histologic type, accounting for ∼90% of patients diagnosed with liver cancer [2]. Infection by hepatitis B and C viruses is the main risk factor for HCC, and nonalcoholic fatty liver disease (NAFLD) is becoming a growing cause of HCC in the United States [3, 4]. Although advancements have been made in treatment, most patients with HCC present with intermediate and advanced stages of the disease, and treatments are frequently not curative [5, 6]. Prediction of clinical outcomes is being challenged because of the insidious symptoms and the high heterogeneity of HCC. Therefore, developing novel prognostic models for the personalized evaluation of cancer risk is urgently needed.

A recent study published in *Science* found that copper could directly bind to lipoylated mitochondrial enzymes, resulting in proteotoxic stress and destabilization of iron-sulfur (Fe-S) cluster proteins, which leads to cell death [7]. Copper toxicity induces a unique type of cell death distinct from regulated cell death (RCD) (e.g., apoptosis, ferroptosis [8], pyroptosis, and necroptosis [9]). Tsvetkov et al. termed this previously uncharacterized cell death “cuproptosis” [11] and identified several genes that related to copper-induced cell killing. For example, FDX1 encodes a small iron-sulfur protein acting as a mitochondrial reductase and is a direct target of elesclomol [11]. High-level copper concentrations have been detailed in the tumors or serum of patients with cancers, including lung [12, 13], breast [14], gastrointestinal [15], oral [16], thyroid [17], gall bladder [18], and prostate [19] cancers. Copper is crucial for regulating the activity of the autophagic kinases ULK1/2 to promote tumor development in lung cancer [20]. Gunjan et al. reported a case of neurological Wilson's disease developing decompensated cirrhosis and HCC due to copper accumulation [21]. Additionally, copper chelators and ionophores have been suggested as antitumorigenic drugs [22]. Cen et al. reported that disulfiram reacts with Cu to form the Cu complex, which is the active agent that induces apoptosis in human melanoma cells [23]. Cui et al. demonstrated that copper-depleting nanoparticle administration inhibits tumor growth and substantially improves survival in mouse models of triple-negative breast cancer [24]. In the liver, lacking functional ATP7B leads to copper overload, which affects lipid metabolism and cell cycle [25, 26]. The significance of cuproptosis in HCC prognosis and immune function has not been explored.

Most encoding protein RNAs are modulated by one or more miRNAs [27, 28]. MicroRNAs (miRNA) are important in posttranslational regulation of gene expression via binding to messenger RNA, whereas their dysfunction has been demonstrated to mark many diseases including HCC [29]. In this study, differentially expressed miRNAs targeting cuproptosis-related genes (CRGs) between tumor and matched normal tissues of HCC were identified. Using univariate Cox regression and least absolute shrinkage and selection operator (LASSO) penalty, a prognostic cuproptosis-related miRNA (CRM) signature was constructed. The independent prognostic role of the model was determined by applying multivariate Cox regression and its relationship with tumor-immune microenvironment was also investigated. Then, a nomogram comprising the cuproptosis-miRNA signature and clinical variables was also established. Finally, differentially expressed genes (DEGs) based on risk score and immune score were further identified, and functional analysis and immune-related analysis were conducted to explore the potential mechanism.

## 2. Materials and Methods

### 2.1. Data Collection

The expression data of RNA and related information of 374 patients with liver cancer were downloaded from the TCGA database. From the TCGA-LIHC cohort, 184 tumor samples were randomly selected to form a test set. miRNAs targeting CRGs were acquired from the TargetScanHuman database. The transcriptome expression data were normalized utilizing the “limma” package and obtained by the “TCGAbiolinks” package. The acquisition of all data was analyzed complying with TCGA and TargetScanHuman data access policies. Thirteen CRGs were found in the published literature [7] (Supplement Table 1).

### 2.2. Establishment of the Prognostic Cuproptosis-Related miRNA Signature

The differentially expressed CRMs (DE-CRMs) were analyzed by “edgeR” package. Heatmap and volcano plot was used to visualize DE-CRMs. The criteria for selecting DE-miRNAs were log2fold change (|log2FC|)>1 and false discovery rate (FDR)<0.05. Univariate Cox analysis was performed to screen the DE-CRMs with the prognostic value (*p* < 0.05). LASSO analysis was employed for those DE-CRMs to minimize overfitting via “glmnet” package with 10-fold cross-validation [30]. Finally, 14 cuproptosis-related miRNA model and their coefficients were identified for further study. A risk score was calculated using the formula: risk score=∑_*i*=1_^*n*^*βi* × Exp*i* (*β*_i_: the expression level of each miRNA, Exp_i_: Cox regression coefficient of miRNA). The patients with HCC were separated into two risk subgroups following the median risk score. “Survminer” R package was used to perform survival analysis. By using “survival” and “timeROC” R packages, the area under the curve (AUC) gained from the time-dependent receiver operating characteristic (ROC) analysis was measured. Multivariate Cox regression was conducted to test whether the CRM signature was an independent prognostic factor. In addition, survival analysis based on the test set and clinical subgroups were performed to validate the robustness of this risk model.

### 2.3. Development of a Predictive Nomogram

To calculate the probability of 1-, 3-, and 5-year OS for patients with HCC, a novel nomogram was built through “rms” and “regplot” packages. Gender, age, pathological stage, N stage, M stage, and risk score were enrolled in this nomogram. Calibration curves were displayed to estimate the prognostic ability of this prediction model compared to actual survival rates.

### 2.4. GSEA, Immune Cell Infiltration Analysis, and Drug Sensitivity Analysis

To clarify the intrinsic mechanisms of the cuproptosis-related miRNAs, GSEA analysis was performed to compare the biological conditions of the two risk groups. We estimated the correlation of immune cells and related pathways in low- and high-risk patients by applying single-sample gene set enrichment analysis (ssGSEA) with “gsva” R package [31]. The analyses of TIMER, CIBERSORT, CIBERSORTABS, XCELL, QUANTISEQ, EPIC, and MCP counter were implemented to discover the association between immune infiltration and the risk model. In addition, we also explored the relationship between immune checkpoint genes [32] (Supplement Table 2) and the risk model to predict the potential response to immune checkpoint blockade (ICB) therapies.

### 2.5. Identification and Functional Enrichment Analysis of DEGs Based on Risk Score and Immune Score

Risk-related DEGs between the high-risk and low-risk groups in patients with HCC were identified using “edgeR” package. Immune scores derived from ESTIMATE represent the level of infiltration of immune cells in tumor tissues [33]. According to the immune scores, patients with HCC were classified into two groups: high-immune group and low-immune group, and immune-related DEGs were obtained following the immune score. The common DEGs based on risk score and immune score were visualized by Venn diagram. “ggplot2,” “enrichplot,” and “clusterProfiler” R packages were used to perform gene ontology (GO), the Kyoto Encyclopedia of Genes and Genomes (KEGG) analysis was also conducted for DEGs mentioned above.

### 2.6. Statistical Analysis

Statistical analyses were executed with R software (version 4.1.3). Chi-square test was applied to match the categorical variables between the high- and low-risk groups. Student's *t* test was used to compare the continuous variables between the two groups. *P* < 0.05 was considered the cutoff criterion of statistical significance. Adjusted *P* values were achieved by Benjamini and Hochberg (BH) correction.

## 3. Results

### 3.1. Identification of DE Cuproptosis-Related miRNAs

A flowchart of data collection and analyses is described in Figure 1. The gene expression of 374 HCC samples was downloaded from the TCGA database with clinicopathological characteristics (Table 1). miRNAs targeting CRGs were achieved from the TargetScanHuman database. A total of 134 cuproptosis-related miRNAs were differentially expressed between tumor tissues and nontumor tissues. Among them, 117 miRNAs significantly were upregulated in the tumor tissues, whereas 17 miRNAs were downregulated (Figures 2(a) and 2(b)).

### 3.2. Construction of a Prognostic CRM Signature in TCGA Cohort

Nineteen of DE cuproptosis-related miRNAs (DE-CRMs) related to OS were identified by performing univariate Cox regression analysis (Figure 2(c)). To minimize potential overfitting, 19 of DE-CRMs were submitted to LASSO Cox regression analysis to build the prognostic signature. The LASSO coefficients of the 19 survival-related CRMs are illustrated in Figure 2(d). Fourteen miRNAs are included with the best performance of the prognostic model in Figure 2(e). Finally, 14 prognostic cuproptosis-related miRNAs stood out for the establishment of the prognostic model. The corresponding risk scores were computed for the TCGA datasets using multivariate Cox regression analysis (Figure 2(f)), according to the following formula: risk score=e (0.050 *∗* expression level of miR-767-5p+0.177 *∗* expression level of miR-5003-3p+0.055 *∗* expression level of miR-137-3p+0.035 *∗* expression level of miR-760+0.068 *∗* expression level of miR-548f-3p+0.132 *∗* expression level of miR-3171+0.174 *∗* expression level of miR-3189-3p+0.208 *∗* expression level of miR-3620-3p+0.224 *∗* expression level of miR-3911+(−0.537) *∗* expression level of miR-6764-5p+0.187 *∗* expression level of miR-4652-3p+0.246 *∗* expression level of miR-504-3p + 0.068 *∗* expression level of miR-892a +0.336 *∗* expression level of miR-548aq-5p).

According to the median cutoff value, the patients were divided into a high-risk group (n=182) and a low-risk group (n=183). The distributions of the risk scores and survival status supported the classification of patients with HCC into two groups by the miRNA risk model (Figure 3(a)). The differential expression of 14 CRMs between high-risk group and low-risk group is shown in Figure 3(b). The Kaplan-Meier survival curves indicated that the risk stratification could represent the different survival status of patients with HCC. High-risk subgroup exhibited prominently poorer OS relative to the low-risk subgroup (Figure 3(c), *p* < 0.001). Analysis of a time-dependent ROC and AUC found that the prognostic ability of the miRNA model was 0.709 (1 year), 0.712 (3 years), and 0.729 (5 years), which revealed that this risk signature has an accurate predictive ability for the outcome of patients with HCC (Figure 3(d)).

### 3.3. Independent Prognostic Value of CRM Signature and Construction of a Novel Nomogram for HCC Prognosis

Univariate Cox regression analysis indicated that the risk score had important association with OS in TCGA cohorts (*p* < 0.01, hazard ratio [HR]=1.995, 95% confidence interval [CI]=1.253–3.176), as well as several clinicopathological parameters, including pathologic overall stage (*p* < 0.0001, HR=2.993, 95% CI=1.897–4.723), pathological M stage (*p*=0.019, HR=3.991, 95% CI=1.251–12.733). No obvious relevance was caught between clinical parameters and OS of patients with HCC, such as gender, age, and pathological N stage. Multivariate Cox regression analysis supported that risk score is an independent prognostic predictor (*p* < 0.05, HR=1.821, 95% CI=1.126–2.943), as shown in Figures 3(e) and 3(f).

A nomogram was established to serve as a dependable, efficient tool for the prediction of OS in HCC that integrated the miRNA risk signature with significant clinical variables, including age, gender, overall stage, N stage, and M stage (Figure 3(g)). The nomogram could provide the accurate prediction of survival rate in patients with HCC, as shown by the calibration curves (Figure 3(h)). These results implied that the nomogram could act as a quantitative method for the prognosis of patients with HCC and had great significance in clinical practice.

### 3.4. Validation of the Robustness of the CRM Model

To verify the predictive ability of CRM signature, a risk score was calculated for each sample in the test set. The distributions of the risk scores and survival status in test set proved the robustness of this model for stratifying patients with different risk (Figure 4(a)). The expression of 14 CRMs between high- and low-risk subgroups in test set is shown in Figure 4(b). The result of survival analysis indicated the significant differences of prognosis in two risk groups of the test set (*p* < 0.001) (Figure 4(c)). Analysis of a time-dependent ROC and AUC assessed the predictive accuracy of the miRNA model in test set: 0.753 (−1 year), 0.772 (−3 years), and 0.765 (−5 years) (Figure 4(d)). Stratified prognostic analyses were performed based on patient clinical characteristics, including age, histologic grade, overall stage, and T stage (Figure 4(e)). The results showed that cuproptosis-related miRNA signature could distinguish the prognosis of patients at high and low risks in different subgroups.

### 3.5. GSEA, Immune Cell Infiltration Analysis, and Drug Sensitivity Analysis

The result of GSEA revealed that the high-risk subtype enriched in several pathways related to infection and inflammation, which implied that the cuproptosis-related miRNAs might have regulative effects on the activity of inflammation in HCC. Interestingly, signaling pathways were enriched in the high-risk group: NOD-like receptor signaling pathway and Ras signaling pathway, which has been widely studied in association with cancer (Figure 5). To apprehend the implication of miRNA risk status and tumor microenvironment, the infiltration levels of immune cells between high-risk group and low-risk group in HCC were quantified. The heatmap depicted the distinction of immune cell infiltration status in two different risk groups (Figure 6(a)). The infiltration of 16 immune cells and 13 immune-related functions in HCC samples was analyzed with “ssGESA.” Correlations of the ratio of infiltrating immune cells and related functions are shown in Figures 6(b) and 6(c). CD8+ T cells were positively correlated with tumor-infiltrating lymphocytes (TIL), as for immune function, a significantly positive correlation was observed between T-cell coinhibition and check point. To further investigate the effect of immune checkpoint blockade (ICB) therapies, the association between the expression level of immune checkpoint genes (ICGs) and the risk score was also analyzed. Several ICGs were differentially expressed between two risk groups. It is noteworthy that TNFSF9, TNFRSF4, LGALS9, CTLA4, and CD276 were highly expressed in the high-risk group, which demonstrated potential effectiveness of ICB therapy (Figure 6(d)). These data suggest that the signature can predict the response to clinical treatment and may differentiate HCC patients who benefit from treatment.

### 3.6. Identification and Functional Analysis of DEGs Based on Risk Score and Immune Score

Given the important association between immune status and risk score mentioned above, intersected DEGs were also identified and further conducted the functional analysis. A total of 1335 DEGs were identified based on the risk score in patients with HCC, including 988 upregulated genes and 347 downregulated genes (|log2FC| > 1 and FDR < 0.05). Simultaneously, 2023 DEGs were obtained from the immune subgroups. Finally, 581 DEGs both in the risk group and immune group were identified (Figure 7(a)). Functional enrichment analyses were performed to characterize the biological functions and pathways of DEGs. GO functional analysis of the DEGs revealed that they were enriched in biological processes including regulation of hormone secretion, signal release, and digestion, and involved in the component of the synaptic membrane. DEGs were also strongly linked to receptor ligand activity and signaling receptor activator activity (Figure 7(b)). Aberrant signaling processes induce a variety of cancers, and the enrichment in signaling activities uncovered the clinical significance of DEGs. KEGG analysis showed that DEGs were active in neuroactive ligand-receptor interaction, chemical carcinogenesis-receptor activation, and calcium signaling pathway (Figure 7(c)). The results indicated that these DEGs might be thought important to HCC progression.

## 4. Discussion

HCC is one of the deadliest malignant tumors with worse survival rate and high-level heterogeneity. The pathological evaluation and AJCC TNM stage remain the major diagnostic and prognostic methods for patients with HCC, which are not accurate and sensitive enough. Patients with HCC with the same pathological stage have different treatment effectiveness and clinical outcomes. An accurate prediction of prognosis improves the doctors' ability to decide individual treatment strategies by identifying the risk status of patients. Therefore, exploring novel molecular biomarkers is urgently needed for improving the prognosis and quality of life of patients.

Recently, a study by Tsvetkov et al. was published in *Science* and declared a novel form of copper-induced cell death termed cuproptosis [7], which has drawn much attention. Cell death has gained increasing prominence in tumor research, including apoptosis [34], ferroptosis [8], pyroptosis [35], and necroptosis [36]. Moreover, ionophores for copper replenishment can induce cuproptosis. On the other approach for cancer, copper depletion could reduce the activity of angiogenic factors to suppress blood vessel development, and copper chelation has been recommended for cancer treatment due to its role as an antiangiogenic factor [37]. These findings suggested that therapies targeting cuproptosis might be a potential strategy for cancer. However, the value of cuproptosis in cancer prognosis especially in HCC remains unclear. miRNA is a small ∼20–24 nucleotides molecules acting as essential regulators in the development of cancer, which influences cell cycle, metastasis, metabolism, and cell death. miRNAs were frequently found dysregulated in human malignancies and were potential biomarkers for multiple cancers [38, 39]. Especially, prognostic miRNA signatures targeting CRGs have not yet been explored in HCC.

In this study, the expression of miRNAs targeting 13 CRGs in HCC tumor tissues was systematically investigated, and the findings revealed that 19 miRNAs had prognostic value in patients with HCC. Then, a prognostic signature with 14 miRNAs targeting CRGs was constructed, which was proven as an independent predictor by using multivariate Cox regression analysis. Verification by sampling and stratified prognostic analyses exhibited that the miRNA signature has good performance in the prediction of patients' outcomes in HCC. A novel nomogram integrating the risk signature and clinical parameters to provide individualized predictions was also built. Agreeably, the nomogram accurately predicts the 1-, 3-, and 5-year survival rates for patients with HCC. Moreover, different immune infiltrating conditions of the two risk groups were identified to investigate the association between the risk signature and the immune microenvironment. The results demonstrated that risk stratification was associated with several kinds of immune cell infiltration. The immune cells mediated the antitumor immune responses, and dysregulated antitumor immunity was associated with tumorigenesis, progression, and invasion [40]. However, the high-risk subtype was characterized by a distinct infiltration landscape of immune cells compared with low-risk subtype (macrophage, B cells, T cells), speculating that poor prognosis may be explained by the unfavorable immune microenvironment and deficiency of immunomodulation. Finally, the DEGs considering both the risk score and immune score were identified. The results of GO and KEGG revealed that these DEGs were involved in signaling and chemical carcinogenesis-receptor activation that might promote HCC progression. According to the results of GSEA, several signaling pathways also stood out in the high-risk group. Given the importance of the signaling pathways in tumor progression and development, the remarkable significance of this model in discriminating the different risk status was suggested.

Most of the miRNAs in this signature have emerged in studies related to cancers. MiR-767-5p promoted tumor aggressiveness and could be sponged by LINC-PINT in thyroid cancer [41]. Elevated expression of miR-767-5p was found in melanoma tissues and it acted as tumor promotor in melanoma [42]. Upregulated miR-767-5p was associated with cell proliferation, migration, and invasion, revealing the oncogenic role of miR-767-5p in breast cancer [43]. MiR-5003-3p promoted metastasis by targeting epithelial-mesenchymal transition (EMT) regulators in breast cancer [44] and exhibited similar functions in activating tumor progression in gastric cancer [45]. Hu et al. identified miR-504 as a directly suppressive regulator of p53 [46]. MiR-504 regulates ribosomal biogenesis and supports cancer cell survival [47]. Studies demonstrated that MiR-3171 is abnormally increased in bladder cancer and HCC tissues [48, 49]. Overall, these literature indicated that the cuproptosis-related miRNA signature might correlate with HCC progression and revealed prospective targets for the treatment of HCC.

This study has several strengths. It is the first to construct a prognostic signature focused on the cuproptosis-related miRNAs in HCC, which performed well in the prediction of patients with HCC. Second, immune cell infiltration analysis revealed that the miRNA signature existed dysregulated immune functions and the expression profiles of ICGs in different risk groups might provide a therapeutic strategy related to immune checkpoint inhibitors for patients with HCC. A composite prognostic nomogram was also established, and the calibration curve results suggested that the prediction of our nomogram was accurate and reliable. Furthermore, the DEGs based on risk score and immune score were identified to delineate a distinct set of genes. Functional enrichment analysis showed that these DEGs were enriched in some pathways associated with tumor progression. Nevertheless, the limitations of this study incorporate an insufficient sample size and a lack of experimental validation. The profound mechanism of cuproptosis-related miRNAs in the role of immune microenvironment and tumor progression of HCC requires further assessment.

## 5. Conclusion

This study identified a reliable prognostic signature based on cuproptosis-related miRNAs. It acts as a reliable prognostic model, and a nomogram with high availability including the risk score signature was constructed. Our findings might favor personalized prediction and therapeutic strategies. More large-sample studies are demanded to verify the feasibility of the risk signature. The underlying mechanisms between the miRNA signature and the development of HCC warrant further investigation.

## Figures and Tables

**Figure 1:** Flow diagram of data processing and analyses.

**Figure 2:** Construction of prognostic CRM signature in TCGA cohort. Heatmap (a) and a volcano plot (b) of the DE-CRMs in the TCGA cohort; the (c) forest plot of the univariate Cox regression analysis with DE-CRMs; (d) LASSO coefficient profiles of the 19 survival-related CRMs; (e) construction of the cuproptosis-related miRNA signatures by LASSO Cox analysis. The optimal parameter (lambda) was selected as the first black dotted line indicated; (f) forest plot of the multivariate Cox regression analysis with 14 CRMs.

**Figure 3:** Characteristics of the risk score and a nomogram predicting OS for HCC patients in TCGA cohort. (a) The distributions of the risk scores and survival status in TCGA cohort; (b) the expression of 14 CRMs in two risk groups; (c)Kaplan-Meier curves of the miRNA signature in TCGA cohort; (d) the ROC analysis to estimate the predictive efficiency; forest plots of the (e) univariate and (f) multivariate Cox regression analyses in TCGA cohort; (g) the nomogram was constructed based on prognostic signature and clinical variables; (h) the calibration curve for evaluating the accuracy of the nomogram model.

**Figure 4:** Validation of the robustness of the CRM model. (a) The distributions of the risk scores and survival status in test set; (b) the expression of 14 CRMs between two risk groups in test set; (c) Kaplan-Meier curves of the miRNA signature in test set; (d) the ROC analysis to estimate the predictive efficiency of the miRNA signature in test set; (e) subgroup Kaplan-Meier survival analysis.

**Figure 5:** GSEA analysis of TCGA-LIHC.

**Figure 6:** Immune-related analyses. (a) Heatmap of infiltrating profile of immune cells; the correlation between tumor-infiltrating immune cells (b) and related pathways (c); (d) the expression of CD276, CTLA4, LGALS9, TNFRSF8, TNFSF9, and TNFRSF4 between the high-risk and low-risk groups.

**Figure 7:** Enrichment analysis for DEGs. (a) Venn diagram showing the common DEGs based on risk score and immune score; (b) GO enrichment analysis of DEGs; (c) KEGG enrichment analysis of DEGs.

**Table 1:** Clinicopathological parameters of patients with HCC.

Characteristics	No. of patients	Median OS (year)
Age (years)		
<60	172 (45.6%)	1.55
≥60	204 (54.1%)	1.73
NA	1 (0.3%)	—

Gender		
Female	122 (32.4%)	1.73
Male	255 (67.6%)	1.58

Histologic grade		
G1	55 (14.6%)	1.90
G2	180 (47.8%)	1.59
G3	124 (32.9%)	1.58
G4	13 (3.4%)	1.55
NA	5 (1.3%)	—

Pathological stage		
I	175 (46.4%)	1.75
II	87 (23.1%)	1.56
III	86 (22.8%)	1.14
IV	5 (1.3%)	0.61
NA	24 (6.4%)	—

T		
T1	185 (49.1%)	1.75
T2	95 (25.2%)	1.65
T3	81 (21.5%)	1.12
T4	13 (3.4%)	1.39
NA	3 (0.8%)	—

N		
N0	257 (68.2%)	1.63
N1-2	4 (1.1%)	1.79
NA	116 (30.7%)	—

M		
M0	272 (72.1%)	1.62
M1	4 (1.1%)	1.07
NA	101 (26.8%)	—

T: tumor; N: node; M: metastasis; OS: overall survival; NA: not available.

## Data Availability

The datasets presented in this study can be found in online repositories. The names of the repository/repositories and accession number(s) can be found in the article.

## Supplementary Materials

Supplementary Materials Supplement Table 1: Cuproptosis-related genes. Supplement Table 2: Immune checkpoint-related genes.
